# Design of a Real-Time Monitoring System for Smoke and Dust in Thermal Power Plants Based on Improved Genetic Algorithm

**DOI:** 10.1155/2021/7212567

**Published:** 2021-07-01

**Authors:** Bo Wang, Xuliang Yao, Yongqing Jiang, Chao Sun, Mohammad Shabaz

**Affiliations:** ^1^College of Intelligent Systems Science and Engineering, Harbin Engineering University, Harbin 150000, China; ^2^School of Measurement and Communication Engineering, Harbin University of Science and Technology, Harbin 150000, China; ^3^Arba Minch University, Arba Minch, Ethiopia; ^4^School of Computer Science Engineering, Lovely Professional University, Phagwara, India

## Abstract

The major health hazards from smoke and dust are due to microscopic fine particles present in smoke as well as in dust. These fine particles, which are microscopic in nature, can penetrate into human lungs and give rise to a range of health problems such as irritation in eyes, a runny nose, throat infection, and chronic cardiac and lung diseases. There is a need to device such mechanisms that can monitor smoke in thermal power plants for timely control of smoke that can pollute air and affects adversely the people living nearby the plants. In order to solve the problems of low accuracy of monitoring results and long monitoring time in conventional methods, a real-time smoke and dust monitoring system in thermal power plants is proposed, which makes use of modified genetic algorithm (GA). The collection and calibration of various monitoring parameters are accomplished through sampling control. The smoke and dust emission real-time monitoring subsystems are employed for the monitoring in an accurate manner. A dual-channel TCP/IP protocol is used between remote and local controlling modules for secure and speedy communication of the system. The generic GA is improved on the basis of the problem statement, and the linear programming model is used to avoid the defect of code duplication with genetic operations. The experimental results show that the proposed smoke and dust monitoring system can effectively improve the accuracy of the monitoring results and also reduce the time complexity by providing solutions in a faster manner. The significance of the proposed technique is to provide a reliable basis for the smoke and dust emission control of thermal power plants for safeguarding the human health.

## 1. Introduction

The usage of power plants is increasing with the rise in population. To reduce the cost of power generation, to enhance their own competitiveness, to improve the pollution contents, and for corporate benefits, the power generation companies are actively exploring and researching upon the scientific monitoring systems for thermal power plants [1]. However, with the economic development, the environmental pollution problems have become very serious and hazardous for human health. It is essential to protect the environment, to control the pollution, and to ensure the safety of public health by using advanced ecological systems [2–4]. With the continuous stringent requirements of each country on the smoke and dust emission of thermal power plants, the emissions of SO_2_, NOx, and COx in the smoke and dust of thermal power plants have caused great pollution to the atmosphere, so real-time measurement of smoke as well as dust pollutants must be carried out [5, 6].

In [7], the authors designed an online smoke concentration monitoring system based on the filter membrane weighing method. The system uses PLC and WinCC upper computer to control all parts of the system in real time, realizes the requirements of automatic loading of filter membrane, and processes the monitoring data in real time. The system is used to monitor the smoke and dust concentration at the power plant site in real time. The monitoring results show that the system has realized the automatic loading of the filter membrane and the online continuous monitoring which is of great practical significance for various places that require real-time smoke monitoring. However, there is a certain gap between the monitoring result obtained by this method and the actual value, and the reliability of the monitoring result is still to be explored. In [8], the authors have designed a low-cost, high-precision low-concentration smoke and dust detection system. The detection model is based on the theoretical basis of Mie scattering for low-concentration smoke emission requirements. By using the theoretical analysis, a linear relationship between scattered light intensity and smoke density has been determined. The laser emitting unit, signal receiving unit, and STM32 data processing units are designed; the principle of laser modulation has been derived and the weak signal frequency selective amplification principle has also been analyzed. LabVIEW software has been used to write the upper computer program and to display the detection data in real time through the front panel of the computer. The experimental results show that the system has high sensitivity and good scalability and ability to monitor the results online.

In [9], the authors have aimed at the explosion risk of high-concentration combustible dust and, in order to handle this problem, a large-range online dust concentration monitoring system is being designed. The system is based on the principle of light transmission and the dust concentration information. The information regarding dust concentration is collected through the transmitted light signals. The system as a whole contains 6-unit modules to realize the acquisition, conversion, display, and control of signals. Among these 6-unit modules, STM32 is selected as the single-chip microcomputer due to superior performance, and the upper computer program is designed with NI's virtual instrument software. In comparison to a fixed-volume calibration device, the monitoring system proposed in [9] can effectively monitor the dust concentration range of 10–100 g/m^3^ but, beyond this range, the accuracy of the monitoring results is low.

In [10], the authors have aimed at the problems of scattered coalbed methane extraction sites where there are difficulties in real-time communication and collection of production. The authors have used wireless sensor network technology to realize on-site data collection, data transmission, real-time monitoring, and other management tasks. Aiming at the problems of wireless sensor network communication being susceptible to interference, limited communication distance and limited lifespan of wireless sensor nodes have been considered. The usage of CPU, C-MAC protocols, general wireless sensor nodes, wireless gateways, repeaters, and other products based on this technology is promoted. For collecting the data in drainage and mining fields, serial port, parallel port, USB port, and other communication interfaces are configured in the leaf nodes. Redundancy technology and statistics theory algorithms are used to improve the system reliability in the design of background management system. However, this method is designed with sensor networks but it has limitations of long monitoring time.

Traditional smoke and dust monitoring systems are mainly based on laboratory analysis of air extraction and sampling methods [11]. The real-time monitoring of smoke and dust is still a challenging job. In instrumental monitors, optical and electronic technologies such as ultraviolet fluorescence SO_2_ monitors, chemiluminescence NOx monitors, and nondispersive infrared CO_2_ detectors for measuring gas pollution are used. These instruments are usually limited to single-point monitoring and cannot be used at large-scaled organizations [12, 13]. To promote sustainable ecological systems, it is essential to use innovative mechanisms for monitoring smoke and dust particles in the environment [14–21].

In [22], the authors have investigated the saliency detection methods for smoke detection. The performance of the deep saliency network technique (DSNT) has been compared with the existing smoke monitoring techniques. The DSNT method is an end-to-end technique to detect smoke and to predict the existence of the smoke. In [23], the authors have introduced an innovative smoke alarm system based on ZigBee transmission technology (ZTT). The ZTT uses E-charts for visualization of data and random forest to classify smoke. It considers the real-time dynamic environmental factors and produces more accurate results. It is using alarming system for generating the warning for fire in the plants. The user can sense the room environment more intuitively through data visualization E-charts. The proposed ZTT system comprises smoke detection (SD) component, data visualization module, and a wireless communication module. The environmental data is classified into normal air, water mist, fire due to cooking, and fire due to smoke accurately by the proposed ZTT. In [24], a spatial-temporal motion spectrum (STMS) approach based on neural network structure is proposed for extracting smoke features and for evaluating the concentration of smoke more accurately. The usage of LiteFlowNet is explored to ascertain the optical flow from the sequence of an image. Marr-Hildreth technique is explored and merged with this network to eliminate occluded regions from the flow map. An evaluation module is developed using Context-Encoder network for determining smoke concentration levels. Finally, an assessment method is used to evaluate the results of STMS approach with the state-of-the-art models. On the basis of experimental study, the proposed STMS approach provides 97.3% accurate results on specialized datasets taken for research study.

According to the requirements of technical requirements and detection methods for continuous monitoring system of flue gas emission from fixed pollution sources and continuous monitoring of flue gas emission in thermal power plants, the real-time smoke and dust monitoring systems must be explored, which can produce results with better accuracy to stop hazardous impacts of the smoke particles on human health. However, many existing approaches are there as discussed above but still there is a requirement to invent more dynamic smoke detection systems that can monitor smoke and dust particles and alert the humans to take corrective and preventive actions to stop the hazardous impacts of poisonous gases and fine particles which can harm lungs, heart, and other body parts of humans. Based on the improved genetic algorithm, the optimized monitoring system is proposed, which can work on Cloud and can be implemented easily to monitor dust and smoke particles.

## 2. Proposed Real-Time Monitoring System for Smoke and Dust in Thermal Power Plants

With higher restrictions on smoke and dust emissions, traditional smoke and dust monitoring technologies can no longer meet the needs, and the demand for effective smoke and dust monitoring is increasing. Due to the wide variety of pollutant gases in the smoke and the relatively complex chemical reactions in those gases, the monitoring of smoke and dust is a cumbersome task. Hence, this research problem has motivated us to propose a dynamic smoke and dust monitoring system.

### 2.1. System Architecture

The main function of the real-time monitoring system for smoke and dust in thermal power plants is to obtain the concentration of harmful gases and dust in the flue and to assist in monitoring the working conditions of the coal-fired system. There are 8 standard monitoring parameters considered for the research study: 3 pollutant parameters (SO_2_, NOx, and Soot), 3 wet flow parameters (flow rate, temperature, and pressure), and 2 conversion parameters (dry basis oxygen content and emission concentration conversion). The design of the system should consider the openness, low cost, high reliability, and good expansibility. In this research study, an attempt is made to consider all these parameters. The complete monitoring system is able to handle data acquisition and control parameters; multilayer structure is set up as monitoring center with multiple substation systems, and each subsystem can operate independently. The proposed system is named as GA based monitoring system (GAMS).  Figure 1 shows the overall architecture of the proposed monitoring system.

The main program of the system adopts multilayer architecture. The system structure is composed of database server, multiple application servers, web server, and client. It realizes the mode of separating data, control, and operation. It is scalable and hierarchical architecture. The smoke information is generated from geographical data, power load, and power generation information. The next platform in the GAMS framework does the sampling control; it allows the controlled generation of volume of data. The proposed system is applied on the parameters extracted in the database and then provides the real-time information on smoke concentration, harmful gases, and dust particles. The monitoring query is fired after fixed intervals of 30 seconds.

### 2.2. Monitoring System Hardware Subsystem Composition

According to the above working architecture and the technical requirements of the real-time monitoring system of smoke and dust in thermal power plant, the monitoring system is decomposed into several subsystems including sampling control, data processing, monitoring results query, and continuous monitoring of smoke and dust emission. Each subsystem is organized in the form of modules.

#### 2.2.1. Data Processing Module

The main functions of the data processing module are as follows: first of all, obtain the real-time monitoring data measured by the sensor from the serial bus (such as RS232 or RS485 bus), A/D data acquisition card, and other signal transmission conversion media. These data are then transmitted to the data monitoring system for further processing.  Figure 2 shows the basic functional structure of the data processing module.

The analysis of Figure 2 shows that the basic functional structure mainly includes two parts: data collection and data monitoring. The main functions of data monitoring are as follows: first receive the data transmitted by the data acquisition system, and then perform calculation and statistical processing on the obtained monitoring data. Then display the measured data, instrument operating status, and other indicators on the software interface and store the information in the database [16]. In order to meet the requirements of diverse sites and the communication protocols of different environmental protection bureaus, data transmission is designed as independent software so that related functions can be altered at any time.

#### 2.2.2. Sampling Control Module

The sampling control module mainly implements various specific services related to sampling control. It uses the master-slave communication method to communicate with the monitoring instrument through the RS485 small industrial control bus. Through the support of the centralized sampling control mode in the working mode, various functions such as sampling control of the monitoring instrument, failure cause analysis, and maintenance alarm can be realized. It supports I/O sampling and output (e.g., used for monitoring the operating status of pollution control facilities of a pollutant enterprise and can be used to analyze the operating status of its pollution control equipment to find out whether the enterprise has illegally discharged pollutants). It also supports the sampling of A/D conversion (by setting the definition file, can configure the accuracy of A/D sampling, potential drift error, range, conversion coefficient, etc.). Through the combined use of I/O and A/D, it can easily control the work of the monitoring instrument and realize the master/slave working mode in the design. The sampling/control module is a multilayer structured software package that uses JAVA's JNI technology to achieve access to the native API.

Because it is difficult to operate specific hardware in JAVA language, C++ language is used for A/D and I/O operation, and it is packaged into a module that conforms to JNI call interface [18]. For various detection items of multiple monitoring instruments, independent multithreading technology and a system structure serving the critical section of the command queue under multithreading are used to realize the scheduling of concurrent commands. The remote/local control module adopts dual-channel TCP/IP communication means to improve the sensitivity of the system.

#### 2.2.3. Smoke and Dust Emission Real-Time Monitoring Subsystem

The smoke and dust are filtered and diluted by the sampling probe and transported to the corresponding analysis instrument in the control chamber under the flue through the unheated sampling pipeline for continuous monitoring. SO_2_ is analyzed by ultraviolet pulse fluorescence method. Under the excitation of 190∼230 nm ultraviolet light, the SO_2_ gas molecules in the smoke become unstable. When they return to the stable ground state, they will emit fluorescence. The light is measured by a photomultiplier tube. Fluorescence intensity is directly proportional to SO_2_ concentration. NOx is analyzed by chemiluminescence method to measure the NO concentration, and then NO_2_ in NOx is reduced to NO through the molybdenum converter. At this time, the NO signal is subtracted from the NOx signal by the electronic subtractor to obtain the NOx concentration [25]. The continuous monitoring of O_2_ uses the zirconia sensor to analyze the oxygen in the flue gas in real time. When zirconia is heated, due to the migration of oxygen ions in the crystal structure of zirconia, the zirconia crystal becomes a conductive body. The different oxygen concentration in the flue gas makes the current generated by the migration effect different. The circuit diagram of the real-time smoke emission monitoring subsystem is shown in Figure 3.

#### 2.2.4. Monitoring Result Query Module

Data query is meant for the monitoring system to provide data to users. A large amount of historical data is stored in the monitoring result query module, and the data can be updated and maintained in time. Users can query for the data with common characteristics through different query methods. At present, a variety of query methods are provided, including query by city-level administrative region, query by county-level administrative region, query by monitoring time, query by pollution source, and query by pollutant. Multiple query conditions are available for users in each query mode. When the query method is determined, the query condition interface is entered, the query condition can be selected in the interface, and the query result will be displayed in the interface.

According to the design of the above modules, the hardware design part of the real-time monitoring system for smoke and dust in thermal power plants has completed three main functions: First, it can complete the calibration of various monitoring parameters, thereby making the measurement data more accurate; the second part collects real-time data from each hardware module which then processes, stores, and displays the data; the third part sends the field monitoring data to the server of the environmental protection bureau in real time according to the communication protocol formulated by the local environmental protection bureaus to meet the requirements of setting up multiple monitoring systems in diverse sites.

## 3. Implementation of Smoke and Dust Monitoring System in Thermal Power Plant Based on Improved Genetic Algorithm

Based on the hardware design and in order to improve the application performance of the monitoring system, an improved genetic algorithm is used to optimize the design of the system software. The objective function of optimal layout of monitoring points is established, and an improved integer coding genetic algorithm program is developed to solve the optimization model. The characteristics of the algorithm are that the optimized layout of monitoring points has strong pertinence, can avoid the defects of repeated coding after genetic operation, and the genetic solution efficiency is high.

Genetic algorithm is a mature optimization algorithm in the field of artificial intelligence and also an effective tool to solve complex combinatorial optimization problems. However, since the number of monitoring points as optimization variables in this paper has a serial number, the standard genetic algorithm has the defects of repeated coding after crossover, mutation, and other genetic operations in solving combinatorial optimization problems. Many studies have been introduced to repair operators, that is, after each genetic operation; a code duplication check must be carried out to use GA effectively on our problem statement. If duplication is found, the hard repair violates the law of natural genetics, resulting in increase in time complexity of the genetic optimization [26–29]. The improved genetic algorithm is introduced to solve the problem of dynamic monitoring of smoke and dust.

The smoke and dust monitoring system of thermal power plants generally includes two aspects: real-time processing of smoke and dust emissions and environmental restoration after smoke and dust emissions takes place. A linear programming model is established for these two aspects in the following equation:

(1) $$\begin{array}{c} K=\sum_{k=1}^{n}{\left[w_{k}\times \left(x_{jk}-v_{ik}\right)\right]}^{2}. \end{array}$$

In the above equation, *k* represents the type of smoke and dust; *w*_*k*_ represents the treatment time of item *j* smoke and dust. According to actual data regression, it is generally a power function; *v*_*ik*_ represents the treatment effect of smoke and dust pollutants after different treatment schemes; *n* represents the number of monitoring points.

Direct integer coding is used for the monitoring point combination scheme of a chromosome. The advantage is that there is no need for decoding operations. Each integer corresponds to a node number. For example, there are 20 nodes that can install monitoring equipment in a certain area, and 5 of them need to be selected. As a monitoring node, 5 integers are randomly generated in the range of 1–20: 3, 9, 12, 18, and 20 as the monitoring points.

The arrangement of monitoring points should satisfy the following: (a) They should be arranged in a position with higher sensitivity. (b) The monitoring points should be as independent as possible. Based on the above principles and the objective function established according to formula (1), the contribution to a certain failure-prone target value in each monitoring point layout plan is only included in the sensitivity value of the monitoring point with the highest sensitivity. In this way, it is possible to ensure that the optimization results have high sensitivity, and each monitoring point can fully reflect the fault information of different fault points.

First, when there is a nonlinear programming problem with constraints, the objective function of the problem is set as in the following equation:

(2) $$\begin{array}{c} S_{i}=\frac{1}{K-1}\sum_{i=1}^{n}\left(X_{\left(i\right)}-\bar{X}\right){\left(X_{\left(i\right)}-\bar{X}\right)}^{T}. \end{array}$$

In the above equation, *X*_*(i)*_ represents the sensitivity of the measuring point; *T* represents the weight, *K* represents the importance of the node, that is, the possibility of serious smoke pollution.

Calculate the minimum value of the objective function of formula (2):

(3) $$\begin{array}{c} S_{\left(i\right)\min}=\frac{1}{n}\sum_{i=1}^{n}\sum_{j=1}^{m}f_{ij}w_{j}. \end{array}$$

In the above equation, *f*_*ij*_ represents the concentration of smoke and dust; *w*_*j*_ represents the duration of smoke and dust emission.

Crossover and mutation operations are critical optimization steps in genetic algorithms. They not only represent the working principle of the entire genetic algorithm but also determine the final optimization result of the genetic algorithm. The following will introduce in detail the improved crossover and mutation operators introduced to solve the coding duplication problem. When using integer coding genetic algorithm to solve the problem of optimizing the arrangement of smoke and dust monitoring points, each chromosome in the population corresponds to a monitoring point combination plan. Assuming that there are two chromosomes to be crossed, if the traditional single-point crossover method is used (the position of the crossover point is set to 2), the result is shown in Figure 4:

According to Figure 4, there are code duplications in the two chromosomes after crossover. If they are forcibly repaired, they will not only increase the calculation time and amount of calculation but also break the natural evolution of genetic algorithms. Therefore, it is necessary to perform crossover operation. Improve and finally use a fast genetic algorithm to calculate a feasible solution to the problem.

First, the operation process of chromosome ① is as follows: compare the genes before the intersection of chromosome ① with all the genes in chromosome ②; if there is the same gene as ① (the framed part in the figure), then ② will remove the same part, and the rest are in the front row. After the comparison is complete, take out the missing parts in ① from the remaining genes in sequence, and fill in ①. Similarly, the change of chromosome ② is different from chromosome ① but chromosome ② needs to be supplemented with the gene before the intersection point. The chromosomes before and after the improved crossover operation are shown in Figure 5.

According to Figure 5, the above process solves the problem of code duplication after chromosome crossover, which not only avoids increasing the computational complexity of forced repair but also guarantees the natural evolution criterion of genetic algorithm. The calculation flow chart of the integer coding genetic algorithm is shown in Figure 6.

The integer coding genetic algorithm combines mathematics with the biological evolution process based on the biological evolution theory and assumes that the calculation process of the answer to the question is the biological evolution process. It is a new type of calculation method, and its randomness advantage is conducive to complexity. The calculation of questions can accurately and quickly calculate the correct answer. Therefore, this method is often used to solve nonlinear programming problems with constraints, so as to accurately calculate any feasible solution when the objective function of this type of problem reaches the maximum or minimum value, so as to achieve the real-time monitoring.

## 4. Experimental Setup and Result Analysis

The effectiveness of the real-time smoke and dust monitoring system in thermal power plants based on the improved genetic algorithm termed as GAMS system is evaluated along with the benchmarked techniques such as DSNT [22], ZTT [23], and STMS [24]. This section provides highlights of the experimental setup and fine-tuning of parameters.

### 4.1. Experimental Setup and Fine-Tuning of Parameter

Different systems are tested in the same test environment. The test environment is shown in Table 1.

Install the system on the chimney of a 500 t/h boiler, about 60 m above the ground. The smoke and dust sampling system adopts today's advanced dilution sampling method. All analytical instruments are imported from abroad; it is a monitoring system with complete monitoring parameters. The database used in the experiment adopts EDNA real-time database and Oracle large mainstream relational database system, and the application server supports application servers such as Weblogic, Websphere, or Tomcat; the client supports browsers such as IE and Netscape. Because the system adopts a multilayer system B/S architecture, the entire system has strong scalability and easy maintenance and is convenient for safety management. The technical indicators for real-time monitoring of smoke and dust are shown in Table 2.

In order to verify the accuracy of the instrument measurement, the KM940 handheld multicomponent flue gas analyzer from KANE, UK, provided by the Environmental Protection Agency was selected as the comparison instrument. The measurement principle adopted is the constant potential electrolysis method, which meets the national standard HJ/T57-2000's measurement method regulations.

### 4.2. Experimental Results and Analysis

#### 4.2.1. Evaluation of Accuracy of Monitoring Results

The accuracy of monitoring results affects the formulation of smoke and dust emission standards for thermal power plants and has an obvious restrictive effect on the control of smoke and dust emissions. The accuracy comparisons of different methods of smoke and dust monitoring results are shown in Figure 7.

Form Figure 7, the inference can be drawn that, under different iteration times, the accuracy of the state-of-the-art systems is good but the accuracy of the proposed GAMS system for the smoke and dust monitoring of thermal power plants is significantly higher than that of the state-of-the-art systems. The highest accuracy rate of the monitoring results of the GAMS system has reached 97.3%, which outperforms the other benchmarked systems considered for the comparative study. It shows that the GAMS system has obvious advantages in the accuracy of monitoring results and can accurately reflect the status of smoke and dust emission. This proposed GAMS system uses the improved genetic algorithm and establishes the objective function of the optimal layout of monitoring points, making use of the linear programming model, and improved integer coding is employed for improving the GA results and to avoid the defect of repeated coding during genetic operations.

#### 4.2.2. Fitting Analysis of Monitoring Results and Actual Results

In order to further verify the accuracy of the monitoring results of the proposed GAMS system, the smoke emission information of a thermal power plant at different times of the day is collected. The main monitoring objects are SO_2_ and NOx. As a reference, the fitting or variance between the monitoring value of the designed system and the actual value is verified. The results are shown in Figure 8.

From Figure 8, the inference can be drawn that, at different times of the day, the difference between the monitored value and the actual value of the proposed GAMS system is not varying much except certain time instances such as 16:00–18:00 and 12:00–15:00, and certain variance can be seen. The monitoring results of the proposed GAMS method have a least variance between the actual values and the predicted values. The outcome of the monitoring GAMS system is quite satisfactory.

#### 4.2.3. Comparison of Monitoring Time

In addition to the accuracy of monitoring results, monitoring efficiency is also a key indicator to measure the monitoring system. It can reflect the performance of the monitoring system and compare the time-consuming monitoring of different systems. The results are shown in Figure 9.

According to Figure 9, in the initial iteration stage, the smoke and dust monitoring time of the proposed GAMS system is higher than those of the benchmarked existing systems. However, starting from the third iteration, the monitoring time of the proposed GAMS system is significantly reduced and continues to be lower than those of the benchmarked systems. This advantage remains until the end of the iterative test. It shows that the monitoring mechanism of the proposed GAMS system takes lesser time and reduces time complexity by performing faster. It can accurately monitor the smoke and dust of thermal power plants in a short time, which fully illustrates the practical applicability of the proposed system.

The experimental results in this section show that the proposed GAMS system can avoid the defect of code duplication during genetic operations by improving the genetic algorithm. The proposed method is analyzed with respect to aforementioned aspects in this section and it justifies its application and scalable nature. The proposed GAMS monitoring system outperforms the benchmarked techniques.

## 5. Conclusion

With the rapid development of automated systems, network technology, and microelectronics technology in recent years, automated smoke and dust monitoring systems have been designed in order to reduce the negative impact of the hazardous gases on human health. The automated monitoring systems can reduce equipment costs and manual errors and can improve reliability, accuracy, and efficiency of detection systems. The proposed real-time smoke and dust monitoring system is based on a decentralized automated control system, also aiming at economical operations and also being beneficial for common public as it can prevent the thermal plants from spreading poisonous smoke particles in the air. The proposed GAMS system adopts real-time monitoring of the entire power plant's smoke and dust emission information and improves the reliability, efficiency, and efficacy of the monitoring system. The accuracy of the proposed system is recorded as 97.3%, which is a significant milestone in automated monitoring system to detect smoke and dust particles. In order to protect humans from the hazardous impacts of smoke particles, highly accurate automated GAMS system has been designed with six modules, which can be easily integrated in Cloud based, P2P based, and client-server based environment.

## Figures and Tables

**Figure 1:** Schematic diagram of GA based monitoring system (GAMS).

**Figure 2:** Basic functional structure of data processing module.

**Figure 3:** Operation circuit diagram of smoke and dust emission real-time monitoring subsystem.

**Figure 4:** Chromosome situation during standard single-point poor operation.

**Figure 5:** Chromosomes after improved crossover operation.

**Figure 6:** Calculation flow chart of improved genetic algorithm.

**Figure 7:** Comparison of accuracy of monitoring results.

**Figure 8:** The fitting of the monitored value and the actual value. (a) Actual monitoring value; (b) monitoring value of designed system.

**Figure 9:** Comparison of monitoring time between the proposed and benchmarked systems.

**Table 1:** Test environment.

Classification	Project	Parameter
*Hardware environment*	Server	5 units, each with 24 cores
	RAM	16 GB
	Hard disk	2T

*Software environment*	Operating system platform	Linux CentOS
	Server platform	Tomcat
	Database	3 installed EDNA, 2 installed Oracle
	Software platform	Weblogic, Websphere, Tomcat

**Table 2:** Technical indicators for real-time monitoring of smoke and dust.

Parameter	Parameter range
Smoke dynamic pressure	0–1800 Pa
Smoke static pressure	−10 ± 10 kPa
Smoke temperature	0–450°C
Smoke velocity	0–25 m s
Total weight	2.5 kg
Dimensions	480 × 260 × 150 mm
Power consumption	About 45 W

## Data Availability

The data used to support the findings of this study are available upon request.

## References

[1] Igor V., Philippe G., Thierry P. (2018). Characterization of smoke and dust episode over west africa: comparison of merra-2 modeling with multiwavelength mie–Raman lidar observations. *Atmospheric Measurement Techniques*.

[2] Norouzi M., Lehtonen M. (2019). Providing fault ride-through capability of turbo-expander in a thermal power plant. *Energies*.

[3] Matt G. E., Quintana P. J. E., Hoh E., Zakarian J. (2018). A casino goes smoke free: a longitudinal study of secondhand and thirdhand smoke pollution and exposure. *Tobacco Control*.

[4] Moradi M., Chaibakhsh A., Ramezani A. (2018). An intelligent hybrid technique for fault detection and condition monitoring of a thermal power plant. *Applied Mathematical Modelling*.

[5] Chauhan A., De Azevedo S. C., Singh R. P. (2018). Pronounced changes in air quality, atmospheric and meteorological parameters, and strong mixing of smoke associated with a dust event over bakersfield, California. *Environmental Earth Sciences*.

[6] Omelian E., Sankrit R., Helton L. A., Gorti U., Wagner R. M. (2020). Sofia/Forcast observations of r aqr: monitoring the dust emission. *The Astrophysical Journal*.

[7] Deng Z., Cheng Y. Q. (2018). Design of on-line smoke concentration monitoring system based on filter membrane weighing method. *Modern Electronics Technique*.

[8] Sun L. F., Zhang Z. P. (2018). The design of low-concentration dust detection system based on mie scattering theory. *Application of Electronic Technique*.

[9] Zhao X. R., Li Q., Wang W. D., Xu Z. Q., Lu H. R. (2019). Design of on-line monitoring system for dust concentration with large range. *China Measurement & Testing Technology*.

[10] Li F. X., Bian J. L. (2018). Design of real-time monitoring and monitoring system for CBM production based on WSN. *Coal Geology & Exploration*.

[11] Sun Y., Li J., Fu X., Wang H., Li H. (2019). Application research based on improved genetic algorithm in cloud task scheduling. *Journal of Intelligent and Fuzzy Systems*.

[12] Wang Y., Liu S., Wu H., Wang C. (2020). On-demand optimize design of sound-absorbing porous material based on multi-population genetic algorithm. *E-Polymers*.

[13] Fedkin N. M., Li C., Dickerson R. R., Canty T., Krotkov N. A. (2019). Linking improvements in sulfur dioxide emissions to decreasing sulfate wet deposition by combining satellite and surface observations with trajectory analysis. *Atmospheric Environment*.

[14] Coleman M. D., Ellison M., Robinson R. A., Gardiner T. D., Smith T. O. M. (2019). Uncertainty requirements of the european union’s industrial emissions directive for monitoring sulfur dioxide emissions: implications from a blind comparison of sulfate measurements by accredited laboratories. *Journal of the Air and Waste Management Association*.

[15] Zhang B., Zhao G., Huang Y., Yaoyao N. I., Qiu M. (2020). Optimal energy management for series-parallel hybrid electric city bus based on improved genetic algorithm. *Mechanika*.

[16] Mason T. G., Chan K. P., Schooling C. M. (2019). Air quality changes after Hong Kong shipping emission policy: an accountability study. *Chemosphere*.

[17] Singh D., Chhabra A., Singh J. (2013). IMCLA: Performance evaluation of integrated multilevel checkpointing algorithms using checkpointing efficiency. *International Journal of Computing and Digital Systems*.

[18] Dogra A., Kaur A., Shabaz M. (2021). Data collection for classification in IOT and heart disease detection. *Annals of the Romanian Society for Cell Biology*.

[19] Kaur M., Kaur J., Singh D. (2019). A novel framework for drug synergy prediction using differential evolution based multinomial random forest. *International Journal of Advanced Computer Science and Applications*.

[20] Wu C., Hu W., Zhou M., Li S., Jia Y. (2019). Data-driven regionalization for analyzing the spatiotemporal characteristics of air quality in China. *Atmospheric Environment*.

[21] Gao Xu, Yongming Z., Qixing Z. (2019). Video smoke detection based on deep saliency network. *Fire Safety Journal*.

[22] Qin Wu, Jiashuo C., Chuang Z. (2018). Intelligent smoke alarm system with wireless sensor network using ZigBee. *Wireless Communications and Mobile Computing*.

[23] Mi Z., Zhang W., Wu X. (2020). Sniffer-net: quantitative evaluation of smoke in the wild based on spatial-temporal motion spectrum. *Neural Computing & Applications*.

[24] Gomez-Amo J. L., Freile-Aranda M. D., Camarasa J. (2019). Empirical estimates of the radiative impact of an unusually extreme dust and wildfire episode on the performance of a photovoltaic plant in western mediterranean. *Applied Energy*.

[25] Li Y., Ren J. (2017). Study on soft-sensors of boiler flue gas oxygen content based on PSO-lssvm. *Computer Simulation*.

[26] Ba R., Chen C., Yuan J., Song W., Lo S. (2019). Smokenet: satellite smoke scene detection using convolutional neural network with spatial and channel-wise attention. *Remote Sensing*.

[27] Saini G. K., Chouhan H., Kori S. (2021). Recognition of human sentiment from image using machine learning. *Annals of the Romanian Society for Cell Biology*.

[28] Bhola J., Soni S., Cheema G. K. (2020). Genetic algorithm based optimized leach protocol for energy efficient wireless sensor networks. *Journal of Ambient Intelligence and Humanized Computing*.

[29] Yang S., Preiler J., Wiegner M., Lwis S. V., Finger D. C. (2020). Monitoring dust events using Doppler lidar and ceilometer in Iceland. *Atmosphere*.

